# Health Recommendation System using Deep Learning-based Collaborative Filtering

This article has been retracted.

**DOI:** 10.1016/j.heliyon.2023.e22844

**Published:** 2023-11-24

**Authors:** P. Chinnasamy, Wing-Keung Wong, A. Ambeth Raja, Osamah Ibrahim Khalaf, Ajmeera Kiran, J. Chinna Babu

**Affiliations:** a Department of Computer Science and Engineering, MLR Institute of Technology, Hyderabad, India; b Asia University, Taiwan; c PG Department of Computer Science, Thiruthangal Nadar College, Chennai, 600051, India; d Department of Solar, Al-Nahrain Research Center for Renewable Energy, Al-Nahrain University, Jadriya, Baghdad, Iraq; e Department of Computer Science and Engineering, MLR Institute of Technology, Hyderabad, Telangana, 500043, India; f Department of Electronics and Communication Engineering, Annamacharya Institute of Technology and Sciences, Rajampet, AP, India

**Keywords:** Recommendation system, CNN, RBM, Collaborative filtering, Deep learning, Health Recommendation system

## Abstract

The crucial aspect of the medical sector is healthcare in today's modern society. To analyze a massive quantity of medical information, a medical system is necessary to gain additional perspectives and facilitate prediction and diagnosis. This device should be intelligent enough to analyze a patient's state of health through social activities, individual health information, and behavior analysis. The Health Recommendation System (HRS) has become an essential mechanism for medical care. In this sense, efficient healthcare networks are critical for medical decision-making processes. The fundamental purpose is to maintain that sensitive information can be shared only at the right moment while guaranteeing the effectiveness of data, authenticity, security, and legal concerns. As some people use social media to recognize their medical problems, healthcare recommendation systems need to generate findings like diagnosis recommendations, medical insurance, medical passageway-based care strategies, and homeopathic remedies associated with a patient's health status. New studies aimed at the use of vast numbers of health information by integrating multidisciplinary data from various sources are addressed, which also decreases the burden and health care costs. This article presents a recommended intelligent HRS using the deep learning system of the Restricted Boltzmann Machine (RBM)-Coevolutionary Neural Network (CNN) that provides insights on how data mining techniques could be used to introduce an efficient and effective health recommendation systems engine and highlights the pharmaceutical industry's ability to translate from either a conventional scenario towards a more personalized. We developed our proposed system using TensorFlow and Python. We evaluate the suggested method's performance using distinct error quantities compared to alternative methods using the health care dataset. Furthermore, the suggested approach's accuracy, precision, recall, and F-measure were compared with the current methods.

## 1 Introduction

Nowadays, the internet has access to everything. Before making any online purchase, consumers look for product reviews and comments available online. Based on comments, citizens might become frustrated at a certain period as to whether or not that product is preferable. A recommendation algorithm, therefore, offers a forum for recommending an item that is useful and appropriate to individuals. Such a framework is based mainly on product attributes, customer expectations, in addition company information. This filtering-based method progressively gathers a bulky quantity of data via a person's preferences, scores, desires, or actions and instead analyses these details to provide critical information [1,2]. Different methods are designed to extract vast volumes of data effectively. Still, several unordered and unpasteurized files that could be used in numerous configurations must be analyzed. The most potent example of implementing extensive data analysis in multiple areas of functioning is healthcare [3]. Health insurance centers, laboratories, and pharmacies distribute information and reports. The truthfulness of health records is also critical in terms of the three V's. (volume, variety, velocity) by its activities and improve health care coverage [4].

A recommendation scheme has the potential to predict whether or not such a consumer should buy products, dependent mainly on the desires of the customer. This scheme could be applied based on the profiling of a person or the profiling of even an object. This article describes the item-based cooperative filtering-based health advisory program that delivers physicians with helpful knowledge based on a characteristic of an object. Now, there are several internet-accessible websites and authorized users whereby individuals can have viewpoints, feedback, websites, and numerous product perceptions. The recommendation systems system would make decisions concerning customers who may only provide feedback once they obtain input for every item from patients. With the help of a recommendation framework, the popularity of e-business websites was attempting to increase their profit margins throughout the profitable market [1]. Millions of e-commerce users buy products via web pages that interact. Following their purchases, individuals provide reviews or other comments about something else on a related social media platform.

The article's remaining sections are organized as below. An explanation of a collaborative-based filtering recommendation framework is given in section 2. Section 3 discuss the related works of different recommendation system. The theoretical RBM-CNN approach is discussed in section 4. An analysis of various methods with the proposed methodology and hypothetical results is shown in Section 5. The findings and suggestions for future work are discussed in section 6. Finally, we concluded in section 7.

## 2 Background

### 2.1 Preliminaries of recommendation system

Two key factors, especially patients and items, are essential in proposing methods. Patients express desires for specific items, and it is necessary to extract those preferences from the data that has been gathered. The collected data is displayed as a practicality structure, providing the numerical value of each patient-item combination and the degree of that patient's preferences for specific items. Patient-based and item-based recommendation systems are the two categories under which the recommendation mechanisms fall. In a patient-based recommendations system, users provide product ratings and preferences [5]. We can promote an item to a patient based on their commonalities with other patients using a patient-based recommender engine, even if they haven't rated it yet. In an item-based recommender system, predictions about patients are derived from the similarity between things rather than patients. The initial task for prediction in recommendation systems is data collection.

#### 2.1.1 Stages of recommendation system

(1) Data gathering: This stage gathers essential medical information and creates a patient's medical history depending on the characteristics, activities, or services obtained by the patient by the patient. A recommendation system will only operate correctly once a well-defined patient description is created. A recommendation approach is based on observations, like online reviews, implicit feedback, and composite suggestions, that are gathered in varied forms [1].
(2) Training phase: This stage accepts as feedback an evaluation from the previous iteration and incorporates such information using supervised learning [[1], [2], [3]].
(3) Prediction/Recommend Process: Preferential things are recommended for clients throughout this process. Regression analysis validated by design, memory-based, or observed actions of patients through interpretation of information gathered during the data collection procedure.

### 2.2 Classification of filtering techniques

To predict the future, the content-based filtering technique evaluates the qualities and characteristics of things. In the case of document recommenders, content-based filtering is commonly utilized. This method generates a recommendation depending on medical factors, including information about item attributes and the customer's previous purchasing histories. Participants expressed their interests' using rankings, which can be favorable, unfavorable, or neutral. This strategy suggests Positively scored things to the patient [1,2], as shown in Fig. 1.

2. Based on Collaborative:

**Fig. 1:** Types of recommendation systems.1.Based on the content:

The recommender system anticipates unexpected results by constructing a patient-item vector of decisions or interests for items. The patient-item vector is matched with the patient's perceptions and experiences to determine how equivalent their biographies seem. The region is formed by patients diagnosed [6]. Patients who may have never evaluated different activities before are provided recommenders for such items, which leads to positive reviews from physicians in their community. The CF could be utilized in a recommendation system for forecasting or decision support [6].

3. Based on Hybrid:

To determine the reliability and productivity of a recommendation system, this strategy combines the preceding two approaches. The other two methods can be used to implement the hybrid filtering technique [3]: By applying the content-based methods to creating a consolidated recommendation system framework. Then, according to its procedures, this methodology employs several hybrid methods like cascading, weighing, mixing, and switching.

### 2.3 The primary developments of the suggested approach

a. Personalized health recommendations: Deep Learning-based Collaborative Filtering enables the creation of customized health recommendations for individuals. By analyzing users' preferences, behaviors, and health data, the system can suggest tailored health interventions, treatment plans, and lifestyle changes, leading to better health outcomes.
b. Improved patient engagement: These recommendation systems enhance patient engagement by providing relevant and timely health-related content. Patients are more likely to follow medical advice and adopt healthier habits when the information is personalized to their needs and interests.
c. Disease prevention and early detection: Health Recommendation Systems can assist in identifying individuals at risk of certain diseases based on their health data and historical patterns. By proactively recommending preventive measures and early detection strategies, the system can contribute to reducing the prevalence and severity of diseases.
d. In the Proposed system, we have combined the deep learning system of the Restricted Boltzmann Machine (RBM)-Coevolutionary Neural Network (CNN) in order to improve the recommendation of the health care system.
e. Finally, the proposed system performance is compared with the existing methods regarding the accuracy, RMSE, MAE, precision, recall, false positive rate, recall and f-measure.

## 3 Related works

The fundamentals of building and operating a collaborative-based recommendation engine were investigated. Moreover, we examine numerous medical difficulties and design an intelligent health recommender system that gives patients high-quality recommendations. Several phases are taken for designing and analyzing health recommendation systems.

The application of significant data analyses in numerous sectors has risen in tandem with the rapid growth of machine learning and data mining. Big data analytics and its associations have gained distinction and acclaim in medicine. Three V's is a important concept for big data applications. Aside from these three Vs., a fourth V is recognized as veracity (if the information obtained is accurate or reliable), which is critical in medicine. The use of recommender systems in filtering massive datasets and metadata is gaining popularity due to the abundance of unfiltered information and data saturation. A novel HRS is required to enhance the healthcare system and concurrently manage patients with many illnesses. A new HRS is required to strengthen the healthcare system and simultaneously monitor patients with several conditions. Prescriptive modeling underpins the decision support system, which anticipates and implements strategic goods to individuals. This methodology can be used in a variety of situations. Healthcare data is a big data analytics field that can be included in the recommendation engine. The mental well-being collaborative filtering is a judgment system that provides appropriate patient data, including healthcare workers and end-users.

This HRS must be honest and reliable for end clients to participate [[7], [8], [9]]. This HRS (shown in Fig. 2) comprises several sections in which a particular item is prescribed. The training stage, the patient profile processing stage, the sentiment classification phase, the privacy protection phase, and the recommendation system phase are the different phases. First, we must acquire a healthcare dataset to which evidence to inform an identification system will be applied. Collecting and preparing a profile health record (PHR) and client registry is essential to this HRS. As an input for the recommendation systems machine to forecast and suggest medical therapies to customers, PHR is a significant worry. We gather crucial details from a medical record associated with PHR for feature extraction. The information is then classified and stored in a warehouse using a classification technique. The three subs of the recommendation systems process are the data-gathering, training, and content-based recommendation phases. Proper therapies are suggested to patients, and healthcare authorities are encouraged to implement beneficial treatment strategies and increased health therapy after these processes are applied to the client data. The sentiment evaluation process of HRS gathers a patient's viewpoint to make the best medical decision possible. This aids in determining the views of end users on a specific topic. The HRS's security is ensured during the privacy-preserving phase, which ensures that sensitive data is not altered. HRS is significant for providing decisions in innovative healthcare and can benefit stakeholders. A model for diagnosing depressive disorder can be created using fast convolutional neural networks based on region (R–CNN). The produced photographs of persons involved, who will often assist to the evaluation of mental illness, are used to infer feelings using this algorithm for deep learning that distinguishes vector-based material by looking at changes in the orientation of lips and pupils [10]. In Ref. [11], in this article, DLRS: A Deep Learning-based Recommender System employing software-defined networking (SDN) is created for an intelligent healthcare environment. DLSR uses the following stages: A tensor-based dimensionality reduction system has been suggested for eliminating unnecessary dimensions from the acquired data, a decision tree-based categorization scheme is offered for grouping patient queries according to various diseases, and another convolutional neural network-based system is created to make recommendations regarding the patient's health.

**Fig. 2:** The health recommendation system (HRS).

By Aujla et al. [12,13]. Healthcare recommendation mechanisms work this way by offering end users mobile healthcare services that are always available. The development of patient-driven health recommendation systems presents difficulties. The processing of the enormous quantity of data produced by electronic devices and gadgets, flexible network administration for instantaneous information transfer, and a lack of methodologies for expertise compilation are a few of the significant issues. For these explanations, the defined defining networking (SDN)-based DLRS: A Deep Learning Recommender System is built for intelligent healthcare ecosystems in this study. The assessment results demonstrate the suggested scheme's superiority over other competing plans.

Feng et al. [14], Our goal was to develop Pubmender, an academic recommender system that uses an abstract from a work to identify appropriate PubMed journals. The startup space for features in Pubmender was first built using previously trained word2vec. A deep convolutional neural network (CNN) was constructed to produce an abstract representation of abstracts, and a fully connected softmax model was used to suggest the top journals. To create an empirical dataset, we gathered 880,165 papers from 1130 journals via the central repository of PubMed. We contrasted various recommendation models, including CiteSeer, a collaborative filtering-based recommendation mechanism for the Journal of the Association for Computing Machinery (ACM) digital library, and Cavnar-Trenkle on the Microsoft Academic Search (MAS) engine. Compared to MAS, ACM, and CiteSeer, we observed that the accuracy of our system for the top 10 suggestions was 87.0 %, 22.9 %, and 196.0 % higher, respectively.

Mulani et al. [15], These connected device data, when joined with information from additional sources like medical records, nutritional data, and survey data, can be evaluated using tools for large-scale data analysis and given to engines that offer suggestions to produce practical recommendations. The information will be given to the Actor-network, which will then develop a policy for prioritizing a specific action recommendation after being encoded (state) into the suitable format. The critic network receives the action, state pair, and then produces a reward for the effort, state pair. The Actor network's policy is updated using this incentive. The critic network uses a predetermined Expected Reward to learn. As a result, we discover that utilizing Big Data Analytics tools and clever techniques like reinforcement learning and deep learning can significantly enhance recommendation outcomes for the healthcare industry, assisting in the development of fully personalized systems.

Barrera and others [16], Although recommender systems have been implemented in many products, the insurance industry has yet to see the same penetration level due to the sector's unique characteristics. The current study suggests a novel model for recommending occupational hygiene services that combines deep learning-based modeling with methods for natural language processing. The findings of ranking techniques demonstrated that, compared to other models, the model incorporating remembering and generalizing organizations' preferred activities behaved better. These findings significantly impact decision-making since they can enhance business and employee welfare while limiting customer options based on their profiles.

## 4 The proposed health recommendation system

This section outlines the many phases involved in building the suggested recommendation system and explains each use case.

### 4.1 Creation of recommendation system

Numerous innovative strategies are being developed in this field. In this work, we developed a thorough and workable strategy. The software developer begins by creating a research problem, which includes determining the project's goals. A summary of the development's importance follows the research questions. The engineering team will evaluate a practical proposal, including a thorough inspection, cost analysis, and human resources prediction. The organization can proceed to the following stage, the implementation team, once a statement of the problem has been authorized. The group concentrates on the finer points of the initiatives involved. The organization must do a financial feasibility study and demonstrate why the industry is outlay due to the increase in the project cost compared to conventional ones [[17], [18], [19]]. The development team should provide basic information on the problem and previous research and investigation. The schematic design is then executed in Step 3. A set of stages is used to break down the research questions. The correlation and regression or indications are both recognized at the same time. In preparations for business intelligence, the data sources are acknowledged, and the information is recorded, characterized, then converted. A selecting the appropriate infrastructure tools, such as Hadoop and Cloudera, is a critical step 4. Step 5 involves testing and validating the concepts and associated discoveries before presenting them to participants for action. To guarantee reliability, deployment is done in stages with feedback mechanisms built within at each level. Table 1 depicts the many steps of the HRS design approach. The above procedure is depicted in Fig. 3.

**Table 1:** An overview of big data analytics in a medicine recommendation engine context.

Procedure	Definition
Statement	Depending on the “4Vs,” determine the necessity of big data analytics in healthcare.
Problem Statement	What is the issue that is being tried to address? Why would you employ a big data analytics strategy? Preliminary Concepts
Techniques	Data gathering and attribute selection Conversion of data and statistical procedures, such as association, aggregation, categorization, and neural networks, are all examples of analytical approaches.
Deployment	Performance Analysis & Testing

**Fig. 3:** The systematic flow of HRS.

### 4.2 Blueprint of HRS

We need a methodology for collaborating with clients, physicians, therapists, and healthcare experts to create an HRS. The new framework architecture is broken into three sections (data collection, transformation, analysis, and visualization). The first step was to collect. The sources of data for the health system have been divided into two categories: (i) structured data, which would be organized data with an established format, type of data, and architecture, and (ii) Data that is semi-structured has some structure, however, fails to adhere to a data model, allowing for efficient behavioral monitoring of patients with no standard sequence, attribute values, or configuration. Data created by sensing devices, statistics about infectious illnesses, their sensations and diagnostics details, laboratory test results, drug prescriptions, Scan Images, and X-rays illustrate this data. (iii) Semi-structured data: data that does not correspond to a database schema but takes enough structure for patient satisfaction presentation management. (iv) Unstructured data: information with no clear structure, such as medical prescriptions dispensed in different languages, exploring the implications, clinical documentation, etc. Healthcare is an outstanding demonstration of how and why the 3 V's. of data, velocity, variety, and volume, are ingrained in the statistical information they generate. Multiple medical systems, universities, insurance companies, academicians, regulatory agencies, and other entities share massive data. Recommendations, medical evidence, health records, patient information, heart rhythm, biometrics signatures, physician prescriptions, and other information sources are used. A healthcare automating system combines cognitive computing that uses argumentation methodologies and domain-specific information to make suggestions like human specialists. We should first comprehend the many tips, like any other content-based recommendation topic. The various factions include:

Calorie labeling: Producing suggestions to improve nutrition. The doctor may recommend dietary changes to help people recover from medical problems by ensuring they receive the proper nourishment. Recommendations include balancing foods, food swaps, less spicy dishes, or dietary changes.

a) Physical activity: Depending on the client's condition, recommend the type of meditation and exercises the physician would use to recover quickly. The patient may require location, sickness, temperature, and other factors.
b) Diagnosis: Using abnormalities displayed in recent situations, a doctor can prescribe a treatment plan for a patient.
c) Therapy/Pharmaceutical: developing suggestions for various pharmaceutical regimens for a particular condition or physician therapy.

The method of data analysis contributes to the second aspect of the methodology. Health-related suggestions may be produced as a result of the research process. The users who would be using this realm should be discussed beforehand. The system's final beneficiaries are Doctors, scientists, practitioners, and users. In addition to all of these end users, the health recommender system (HRS) can also be advantageous to academics, physicians, and pharmaceuticals. Recommendation systems' ultimate objective is to reduce operational costs. Using a MapReduce-based Hadoop strategy is a part of laboratory techniques. This approach helps physicians identify the best values to diagnose the patient's symptoms and identify the condition they are dealing with while also speeding up diagnostic procedures.

The visualization component is the third and most significant section of the system. This section has elements that impact how suggested products are offered. Visualization and information extraction approaches are applied to communicate actual to the final patients. The most wholesome interests of the organization must be chosen; however, occasionally, conversation criteria come into play when judging a product. Data-driven methodologies use machine learning and statistical techniques to glean conclusions from diverse data. It offers tailored recommendations based on previous learning experiences and trends gleaned from medical studies. Knowledge representation and ML algorithms can be utilized to categorize information sources. The following phases form the foundation of the proposed HRS architecture:

a) Preprocessing
b) Creation of Patient Profile
c) Sentiment Analysis
d) Recommendation Systems
e) Security and Privacy

#### 4.2.1 Preprocessing

Doctors conduct medical trials on patients to identify ailments such as TB, typhoid, and the flu. Doctors need evidence from the model's parameters to investigate and assess various conditions and discover a cure. Furthermore, there has been a notable rise in the caliber of content generated within the medical field. This phase includes the collection and processing of data. Furthermore, the process would be improved if the necessary data-gathering and consolidation instruments were available. The entire method involves gathering patient-relevant data, including statistical characteristics, symptoms, investigations, lab trials, user health records, and actual information via healthcare facilities to increase the recommender's performance.

#### 4.2.2 Creation of Patient Profile

A patient biography is built at this phase for each patient, containing various data. There would be patient data keeping track of each detailed medical history. This record includes data on patients, physicians, hospitalizations, laboratory tests, Computerized tomography, X-rays, and other resources. If the prospective patient is registered, the entire procedure reverts to its initial state and begins with the data acquisition and construction of a new user medical record. The system changes the person's data as needed in the case of an existing user.

#### 4.2.3 Sentiment Analysis

Ensuring the patient understands the entire system—that is, the system has the potential to uphold the protection of personal data—is essential to supporting the patient-based recommendation system for healthcare care. Data taken from individuals, whether or not it contains appropriate health data, is private and, therefore, should not be abused.

#### 4.2.4 Recommendation system

Recommendations can be developed using the principles that are extracted, as well as the physician's circumstances. Individualized advice is administered to patients. Such suggestions may include remedial and preventative actions, explanations of the factors that cause the illness, or an additional course of psychotherapy.

#### 4.2.5 Security and privacy

The HRS calls for mixing varied clinical evidence to strengthen the content-based recommendation quality and advance medicine. Therefore, maintaining a patient's information security is crucial for biomedical studies. The proposed method efficiently protects identity while maintaining the credibility of the information [[20], [21], [22], [23], [24], [25]].

### 4.3 Design techniques for HRS

As depicted in Fig. 4, we want an architecture composed of several technologies that satisfy the industry constraints and particular parameters of different applications. The instruments included in the architecture emphasize the consumer's needs first and ensure that they are satisfied before any other needs. The design process is the first essential technique for creating the structure. It alludes to a participant's active engagement. Patients should participate actively in the new framework construction because their comments can enhance the overall structure and close gaps in the one currently in place. Feedback from either the physician is therefore crucial. Patients should focus on mental well-being concerns while creating recommendation systems rather than global pharmaceutical brand management since these technologies might serve as their administrative assistants in supporting people to deal with pressing issues. The most challenging component is speculating an existing structure to enable widespread client and physician engagement. Without such direct involvement of physicians, various instruments might aid in rehabilitation [[12], [26], [27], [28], [29], [30], [31], [32], [33], [34], [35], [36], [37], [38]].

**Fig. 4:** The health recommendation framework.

The use of differential privacy is the second key instrument for HRS. Cryptography preserves data security, thus addressing the major issue with recommendation systems. In this instance, the exchange of a clinical encounter occurs without compromising the individuals' identification. Therefore, the end client will receive privacy. Patients frequently need the mandate to protect, contrary to their long-term interests. The customers' privacy rights must have been a critical consideration when implementing an efficient health care recommendation system. Differential cognitive factors and degrees of digital skills are tied to technologies since understanding confidentiality hazards on the web is crucial.

Adequate and appropriate communication should be used as the third tool. Reversible communication takes place (to the patient and the recommender). For clinicians to evaluate patients ‘clinical symptoms and provide recommendations for a specific ailment, patients can communicate with doctors in an uninhibited and hardship approach. The goal of the recommender system should be addressed by visualization techniques, which should also be able to comprehend the patient, doctors, and their intents.

### 4.4 Evaluations of HRS

The criteria for judging the classification method must be carefully chosen to ensure the program's effectiveness. Traditionally, information-gathering parameters were used to analyze decision support systems [23,39]. Typical metrics considered in the assessment include:

i. Precision: The percentage of relevant items that are found when searching which is shown in equation (1).

(1) Precision=TP(TP+FP)

ii. Recall: The percentage of accurately suggested items also included in the list of presented valuable objects which is shown in equation (2).

(2) Recall=TP(TP+FN)

iii. F-Measure: This accuracy measurement plays a role in the quality mean of the study's recall and precision which is shown in equation (3).

(3) FMeasure=(2*Precision*Recall)(Precision+Recall)

iv. The ROC Curve is a tool for comparing diagnostic testing. The actual positive rate and the false positive rate are plotted in this graph. It serves as a metaphor for how overall sensitivity interacts.
v. RSME: This measurement establishes the confidence interval of error variance or the discrepancies among known and correlation coefficients.

To gauge the effectiveness of an HRS depending on medical satisfaction with the services, the content-based recommendation system's assessment methods are crucial. Developing the system fit for specific patients enables it to function by patient needs, allowing the patient not to experience any difficulties and, eventually, improving clinical science.

The professional responsible for developing health recommendation systems should exercise caution and create a plan per regulations. A recommendation system's effectiveness can be evaluated in light of the physician's outward conduct. A service has been developed, and behavioral assessments can determine the system's performance. Keep up with developments, for instance, when assessing patients' medical improvement and making therapeutic interventions. The administration finds it challenging to evaluate the effectiveness of food restrictions for physicians since some people might inhale secretly.

### 4.5 Architecture used for the health recommender system

Finding methods to maintain security and privacy has become crucial as recommendation systems and data mining algorithms are popular. Various privacy issues are raised by customized prescriptions, which may well be successful in drawing in Medicare applicants. According to study findings, confidentiality concerns may induce potential customers to avoid an e-commerce website. Then, whereas the recommendation systems services are being provided, numerous unavoidable security issues emerge that attempt to breach the firewall. In order to address these concerns, this paper will look at a variety of privacy-preserving dependent recommendation engines, including the approach used by deep learning, SVD, etc., from which the algorithm can generate recommendations without access to client assessments.

#### 4.5.1 Auto-encoder-equipped perceptron with multiple layers

This feed-forward neural network employs a recurrent neural network with an adjustable convolution operation and includes numerous hidden units. Unsupervised machine learning is the foundation of the auto-encoder (AE), which seeks to refabricate the input data in the output. Fig. 5 illustrates how an auto-encoding neural network uses the backward propagation algorithm for learning to figure out how to elevate the error message using the proper neural network parameters. The brains of feature representation can be conceived of as auto-encoders.

**Fig. 5:** Neural network based on Auto Encoder.

Compression algorithms, data reconstructing for unsupervised learning, and principal component analysis typically encode information by splitting big matrices into shorter matrices that preserve the matrices' most essential attributes.

### 4.6 The working of proposed health recommendation system using RBM-CNN

All elements seen are connected to all aspects hidden by different indicators in the normal RBM. Given how big the frames are, using an RBM to recover spatial information from entire structures for object classification is not encouraging—an RBM modeling version known as the convolutional RBM was developed to address this issue (CRBM). The CRBM is a two different model, like the RBM, wherein the concealed and apparent independent variables are organized as matrices. As a result, both suppressed and noticeable units can define proximity and neighborhood in this paradigm. The viewable matrices of the CRBM may depict a visual, and its sub-windows may depict individual image overlays. The hidden-visible interconnections in the CRBM are local, and values are distributed among hidden layer groups. As a result, CRBM is superior to RBM and CNN because it takes advantage of both of their capabilities.

a) Since files do not carry labels, upload the medical dataset while simultaneously setting pass header = none.
b) The evaluation dataset should be loaded. Then, modify our fields in such frames so that we will all communicate data effectively. Confirm the data sets' modifications.
c) Data cleansing and modification and compare the number of hospitals with evaluations according to hospital ID.
d) The number of participants is used for instruction and the training list.
i. The PID will be assigned for every participant in the subgroup.
ii. Make a temporary file that holds the ratings for each medical facility.
iii. For each medical service listed in our patient's medical list for no.
iv. Multiply the score by five and include the rankings list in the learning list.
e) Use 15 CNN epochs to train RBM, with a batch size of 100 and 10 for each generation.
f) Following training, the mistake is displayed epoch by epoch. Choose the supplied physician.
g) It is nourishing the patients and rebuilding the input.
h) List the top 20 institutions for our fictitious patient by ranking the list according to the ratings each received from our model. Analyze the data to determine the pretend patient's Patient ID.
i) Combine the expected ratings from his previous data, including all the clinics our representative participants attended.

## 5 Performance evaluation and discussion

We have conducted our proposed experiment on a healthcare data set [40], which contains 10,000 distinct patient reviews, ranging from 1 to 5, for 500 health facilities. In a proportion of 75:25, development and test data are separated from this collection. Here, the findings are evaluated using a 10-fold cross-validation approach. Tensorflow and Python are used to develop the suggested CRBM approach. With several techniques, the HRS was designed and evaluated on a healthcare dataset of evaluation and specific details. We must select K as the number of closest neighbors. The dataset might lose valuable information if K were very small, while its confidential information would be compromised if K were too large. However, it is essential to choose parameter K appropriately. Therefore, we employ the root mean absolute error (RMSE) method since it is simple to measure and identify, allowing us to quickly construct the recommendation systems system's quality factor. It is used in this essay to demonstrate the effectiveness of the various strategies and their correctness.

According to Fig. 6, the suggested RBM–CNN–based content-based filtering technique's RMSE fluctuates with the parameter K and reaches a faultless value whenever K is equivalent to 10. The precision increases as the market fluctuates—better recommender quality results from this.

**Fig. 6:** The Proposed RMSE values comparison with existing methods.

Table 2 shows the findings for various K values, and for K = 10, the results demonstrate that RBM-CNN performs excellently in RMSE. According to the research observations, the RBM-CNN methodology is the most accurate. RBM-CNN ought to be the favored approach for content-based filtering as a conclusion. Alternative metrics that could be used to evaluate the quality of content-based recommendations include ROC, accuracy, recall, and Mean Absolute Error. Personalized recommendation systems based on deep learning are assessed using different numbers of epochs. As stated in Table 3, each technique is considered using MAE. Fig. 7 demonstrates that the accuracy increases with the number of periods. As a result, the recommendation systems performance is improved.

**Table 2:** Comparison of RMSE values with different methods.

K	MF	SVD	WSVD	RBM	Proposed
5	2.86	2.77	2.74	2.69	2.63
10	2.682	2.69	2.68	2.64	2.56
15	2.71	2.65	2.69	2.65	2.57
20	2.75	2.74	2.74	2.69	2.64
25	2.79	2.77	2.75	2.69	2.67
30	2.82	2.84	2.79	2.76	2.72

**Table 3:** Comparison of the proposed method with different methods based on the number of epochs and MAE values.

No of Epochs	MF	SVD	WSVD	RBM	Proposed
0	0.15	0.16	0.13	0.13	0.11
2	0.086	0.082	0.075	0.069	0.057
4	0.076	0.067	0.062	0.056	0.046
6	0.069	0.059	0.054	0.049	0.036
8	0.066	0.058	0.053	0.046	0.035
10	0.067	0.056	0.051	0.045	0.034
12	0.065	0.055	0.052	0.044	0.033
14	0.063	0.054	0.049	0.042	0.032

**Fig. 7:** The Proposed MAE values comparison with existing methods.

This proposed scheme improves accuracy when two error metrics, such as RMSE and MAE, are considered by comparing and evaluating all the techniques with the anticipated RBM-CNN system. For identifying a clinic for a specific patient, combining an RBM with Convolutional Neural Network enhances the effectiveness of the recommendations. Table 4 demonstrates the False Positive rate of different methods and Table 5 represents the accuracy analysis of different methods.

**Table 4:** The False Positive rate of different methods.

Methods	False Positive Rate
MF	5.15
SVD	5.25
WSVD	6.45
RBM	7.92
Proposed	4.45

**Table 5:** The Accuracy analysis of different methods.

Methods	Accuracy
MF	93.45
SVD	88.25
WSVD	80.15
RBM	92.65
Proposed	94.71

The accuracy and false positive rate are displayed in Fig. 8, Fig. 9, respectively. Based on the earlier data, we note that the proposed approach has the lowest false positive and highest accuracy rates. The results have been improved due to accounting for the evolution of participant states throughout time. In actuality, reducing the false positive rate is essential, but maintaining a high level of accuracy is necessary. The proposed approach was used in the analysis above to record a minimum false positive rate and a boost in accuracy.

**Fig. 8:** The false positive rate analysis of the proposed method.

**Fig. 9:** The accuracy analysis of the proposed method.

Fig. 10, Fig. 11, Fig. 12 show the study of performance's precision, recall, and f-measure metrics. According to these analyses, the suggested method outperforms the current approaches regarding accuracy, recall, and f-measure characteristics by 95 %, 89 %, and 92 %, respectively.

**Fig. 10:** The precision analysis of the proposed method.

**Fig. 11:** The recall analysis of the proposed method against the existing method.

**Fig. 12:** The F-measure analysis of the proposed method against the existing method.

### 5.1 Use cases to predict heart disease prediction

The heart is responsible for flowing blood throughout the body, and various factors can influence how well it functions. The suggested research would compensate for this disease's (i) blood pressure and (ii) cholesterol levels. The patient's cholesterol level aids in determining the severity of heart disease. It also displays the blood pressure level to confirm the likelihood of sickness. Table 6 shows the various blood pressure and cholesterol levels that impact a person's health**.**

**Table 6:** Heart disease predictions.

Cholesterol Levels	
Range of Cholesterol (mg/dL)	Risk of heart disease
90 to <125 mg/dL	Fit (No Disease)
125> to <159 mg/dL	Border Line
160 > to < 189 mg/dL	High
190 mg/dL and above	Very High
Blood Pressure	
Blood Pressure (mm Hg)	Risk Levels
90/60 (Low)	High
120/80 (Normal)	Fit (No Disease)
140/190 (High) Very High	Very High

## 6 Challenges and future directions

Health Recommendation Systems using Deep Learning-based Collaborative Filtering have the potential to revolutionize personalized healthcare by providing tailored recommendations for individuals. However, they also face several challenges including limitations, and hold promising future perspectives:

Challenges:

1. Data Privacy and Security
- Health data is sensitive, and patient information privacy and security are paramount. The challenging task to enhance data privacy with deep learning models.
2. Data Quality
- Healthcare data can be noisy and incomplete, leading to challenges in building accurate recommendation models. Data preprocessing and cleaning are crucial but can be resource-intensive.
3. Cold Start Problem:
- Recommender systems struggle when dealing with new users or items with limited interaction data, which is common in healthcare. Addressing the “cold start” problem is essential.
4. Integration with Electronic Health Records (EHRs):
- Integrating recommendation systems with existing EHRs and healthcare infrastructure is complex and requires interoperability standards.
5. Limited Generalization:
- Models may not generalize well across diverse populations, as healthcare recommendations can be highly personalized based on cultural, genetic, and lifestyle factors.

Future Perspectives:

1. Improved Data Collection:
- Advancements in wearables, IoT devices, and remote monitoring technologies will provide more affluent and more continuous healthcare data, improving the accuracy of recommendations.
2. Federated Learning:
- Federated learning techniques can enable collaborative model training across multiple healthcare institutions while preserving data privacy.
3. Explainable AI:
- Research into explainable AI methods will make it possible to provide transparent and understandable recommendations to healthcare professionals and patients.
4. Adaptive Models:
- Models that adapt and evolve based on individual health changes and preferences will become more prevalent, leading to more dynamic and practical recommendations.
5. Integration with Telehealth:
- Integrating recommendation systems with telehealth platforms can enhance remote patient monitoring and telemedicine services, providing timely interventions and guidance.

In conclusion, Health Recommendation Systems using Deep Learning-based Collaborative Filtering hold great promise in delivering personalized healthcare recommendations. However, they must overcome challenges related to data privacy, ethics, and model interpretability while embracing future opportunities driven by advancements in data collection, AI explainability, and integration with Telehealth.

## 7 Conclusion

The health recommendation system is one of the newest and most popular methods for extracting further details about a patient from medical data. These algorithms use a comparison of patient preferences to identify suggested hospitals. As a result, they are crucial to the medical industry. State-of-the-art solutions must address the security and confidentiality of information problems with CF-based health recommender systems. This article presented a proposed intelligent HRS using the Restricted Boltzmann Machine (RBM)-Coevolutionary Neural Network (CNN), focusing on data mining techniques for efficient and effective health recommendation systems. The pharmaceutical industry can translate from conventional scenarios to more personalized ones. The system was developed using TensorFlow and Python, and its performance was evaluated using error quantities and accuracy, precision, recall, and F-measure. The proposed method clearly shown that, the accuracy was improved compared to existing health recommender systems. The suggested system provides greater MAE and RMSE than the current approaches. Moreover, the system's recall, f-measure, and precision are higher than the current approaches. We intend to refine our algorithm further to deliver enhanced accuracy while maintaining privacy in future releases. In future, they must overcome challenges related to data privacy, ethics, and model interpretability while embracing future opportunities driven by advancements in data collection, AI explainability, and integration with Telehealth.

## Declaration

We acknowledge that Grammarly AI is a widely recognized and reputable writing assistance tool that assists in the identification and correction of grammatical errors, punctuation mistakes, spelling errors, and offers suggestions for improved clarity and conciseness in writing.

## Data availability

Data will be made available on request.

## CRediT authorship contribution statement

**P. Chinnasamy:** Writing - review & editing, Writing - original draft, Data curation, Conceptualization. **Wing-Keung Wong:** Supervision, Funding acquisition. **A. Ambeth Raja:** Writing - review & editing, Supervision, Data curation. **Osamah Ibrahim Khalaf:** Validation, Supervision, Funding acquisition. **Ajmeera Kiran:** Writing - review & editing, Methodology. **J. Chinna Babu:** Supervision.

## Declaration of competing interest

The authors declare the following financial interests/personal relationships which may be considered as potential competing interests:Wing-Keung Wong reports financial support was provided by 10.13039/501100005007Asia University, Taiwan.
